# Association between the Systolic Blood Pressure Trajectory and Risk of Stroke in a Health-Management Population in Jiaozuo, China

**DOI:** 10.1155/2022/7472188

**Published:** 2022-12-28

**Authors:** Jiejie Li, Yanru Zhang, Xiangdong Xie, Guohui Han

**Affiliations:** ^1^School of Medicine, Henan Polytechnic University, Jiaozuo 454000, China; ^2^Department of Neurology, The Second People's Hospital of Jiaozuo (First Affiliated Hospital of Henan Polytechnic University), Jiaozuo 454001, China

## Abstract

The trajectories of systolic blood pressure (SBP) in a screening population in Jiaozuo were examined, and the association between the different types of SBP trajectories and the risk of stroke was evaluated. Data of a fixed cohort population from the Jiaozuo Stroke Prevention and Control Project Management Special Database System that underwent community screening in 2015, 2017, 2019, and 2021 were collected. Ultimately, a total of 1,451 participants who met the inclusion criteria for this study were included in the analysis, which was performed using group trajectory modeling. The baseline SBP for each trajectory subgroup was characterized at follow-up. Kaplan–Meier analysis for each trajectory group was also performed, and the relationship between the SBP trajectory and risk of stroke onset during follow-up was validated using a Cox proportional hazards model. Based on the SBP from 2015 to 2021, this cohort population was divided into three groups based on the trajectory development patterns: the low-stable group (37.6%), the moderate-increasing group (53.4%), and the high-acutely increasing group (9%). Gender, age, body mass index, diastolic blood pressure, and fasting blood glucose level were predictive factors for the SBP trajectory group. The cumulative survival risk in the high-acutely increasing group was higher than that of the other two groups. After adjusting for potential confounding factors and using the low-stable group as a reference, the hazard ratios (95% confidence interval) for the risk of stroke onset in the moderate-increasing and high-acutely increasing groups were 1.38 (0.91–2.07) and 1.51 (0.82–2.76), respectively. The results of the analysis demonstrate that higher blood pressure trajectories are associated with a higher risk of stroke and that the risk of stroke can be reduced by better control and management of the SBP.

## 1. Introduction

Stroke is an acute cerebrovascular disease that includes ischemic stroke and hemorrhagic stroke, among other types, and it refers to a type of disease that causes brain tissue damage due to the sudden rupture or blockage of blood vessels in the brain. Stroke, which has a high incidence rate, high recurrence rate, high disability rate, high mortality rate, and high economic burden, has become one of the most serious diseases that threatens human health. According to the Global Burden of Disease Report (2019), stroke is the second-leading cause of death worldwide after coronary heart disease, accounting for 11.6% of all deaths [1]. At the same time, the increase in the proportion of deaths from stroke has increased the global burden of stroke. According to the Global Stroke Burden, low and middle-income countries exhibit the highest stroke burden. As a developing country, China exhibits a disease burden from stroke that continues to increase, resulting in great pressure on the families of stroke patients and society [2]. The degree of blood pressure control and other risk factors for stroke, as well as the risk of stroke, vary greatly from region to region. According to the Jiaozuo Stroke Prevention and Control Project Management Special Database System, the proportion of the screening population in Jiaozuo City with a high risk for stroke is 21.5%, which demonstrates that the current state of stroke prevention and control in Jiaozuo City is grim. Therefore, investigating the risk of stroke in the population in Jiaozuo City is of great importance.

Hypertension is one of the most common chronic diseases in the world, and it is also considered to be a major risk factor for stroke events [3–5]. From 1991 to 2015, the prevalence of hypertension among Chinese adults continued to increase, with an overall increase of 17.90 percentage points during this period [6]. In both adults and children, the onset of stroke is associated with a high BP level [7–10]. Otherwise, there is evidence that high systolic blood pressure (SBP) ranked first among five other important risk factors for stroke in 2019 [11]. A long-term high SBP can cause lesions in the walls of small arteries, resulting in the stiffening of the lumen and thickening of the intima, which can lead to ischemia and hypoxia in brain tissue when the lumen of the cerebral vessels narrows or becomes occluded. The results of a prospective meta-analysis of 61 populations worldwide (approximately 1 million people) demonstrated a continuous, independent, direct, and positive association between the SBP and stroke risk. The risk of cerebrovascular disease increases twofold for every 20 mmHg increase in the SBP within the range of 115–185 mmHg [12]. Cederholm et al. performed a study that demonstrated an 86% increased risk of stroke in individuals when the SBP was ≥140 mmHg, using a mean SBP of 110–129 mmHg as a reference [13]. Although a high baseline SBP was also determined to be an independent risk factor for stroke, the effect of the SBP trajectory on the stroke outcome was stronger than that of the baseline SBP, which is consistent with the results of the study performed by Portegies et al. [14]. Moreover, the factors influencing the SBP trajectory are essentially the same as those influencing the risk of hypertension. In a recent study of Chinese adults that explored the factors that influence BP trajectories, the participants were divided into three groups based on the SBP trajectory. Among them, an age of ≥40 years, male sex, a BMI of ≥24 kg/m^2^, and Eastern region location were potential factors that influenced the rapid increase in the SBP trajectory and high baseline SBP [15]. In addition, other studies have reported that lifestyle [16], fasting blood glucose level [17], and blood lipid levels [18] are also closely related to the BP level.

A higher SBP is associated with an increased risk of stroke [19]. However, most studies that draw this conclusion are based on a single measurement of the SBP and do not consider the trends in the SBP over time. The SBP increases with age and varies at different life stages. One-time BP values that do not take into account changes in the SBP level are not reliable. Therefore, the results of cross-sectional studies are less accurate than those that consider the trends in the SBP over time [20–22].

Group-based trajectory models are advantageous for analyzing longitudinal data. They assume that the population under study is heterogeneous, that there are multiple groups of trajectories with different potential patterns of development in that population, and that all individuals in each trajectory group have the same or similar trajectories. This type of model is used to describe and characterize the continuous dynamic change in the level of development of a certain thing (such as age) over time, which is different from the information at a specific point in time [23, 24]. SBP trajectories use a group-based trajectory model to describe the dynamic changes in the SBP over time [13]. Currently, group-based trajectory models are widely used in medical research to evaluate disease outcomes over time [25].

In recent years, the impact of SBP trajectories has attracted an increasing amount of attention. One meta-analysis demonstrated that different BP trajectories were associated with different clinical outcomes of stroke, and overall, the lower the BP, the lower the risk of adverse outcomes in these trajectory groups [26]. Multiple studies on the relationship between BP trajectories and clinical outcomes after admission in stroke patients have demonstrated that the low SBP trajectory group generally has a more favorable stroke outcome [27, 28]. Studies analyzing the relationship between BP, stroke, and mortality through SBP trajectories have confirmed that hypertension and rapidly rising SBP patterns are associated with higher risks of stroke and death, whereas moderate hypertension is associated with only an increased risk of stroke. Therefore, monitoring the SBP level and its trajectories is an important part of stroke prevention [14]. Most studies on the relationship between SBP trajectories and stroke have included hospitalized patients, whereas analyses of large-scale health-management populations exploring the risk of stroke are limited.  Table 1 provides a summary of the strengths and challenges of the relevant literature.

This paper is organized as follows.  Section 2 outlines the materials and methods used to collect and process the SBP data.  Section 3 of this paper analyzes the SBP data and presents the results. The results are discussed in Section 4 of this paper.

## 2. Materials and Methods

### 2.1. Data Sources

This study was a retrospective, community-based fixed-population cohort study conducted in Jiaozuo City, Henan Province. In the comprehensive quality control results of the screening and intervention projects for groups with a high risk of stroke in 2020, the single score of the out-of-hospital screening in Jiaozuo ranked first in the country and was tied for third place in the overall country rankings. Before the follow-up of the healthy population, the medical staff were trained by professional physicians and were randomly checked, and the entire follow-up process was standardized under supervision. The data sources used in this study are reliable. This project relies on the National Major Public Health Service Project-Screening and Intervention Project for High-Risk Populations of Stroke, which has been approved by the Jiaozuo Stroke Prevention and Control Center. Data were collected and pooled for the population screened in 2021. Participants came from two representative urban and rural areas, Jiaobei Community and Dafeng Town, Jiaozuo City. In the study, 2,347 individuals participated in 2015, 2,049 individuals in 2017, 2,411 individuals in 2019, and 3,318 individuals in 2021. Participants who dropped out of the stroke screening program or had incomplete data, such as BP and FBG measurements, were excluded. A total of 1,451 participants were finally enrolled in the study.

### 2.2. Data Collection

The entire data collection process was standardized by experienced medical staff, and written informed consent was obtained from the participants. The participant demographics, medical history, BP, FBG level, blood lipid levels, and other variables were sequentially measured. Demographic data on gender, age, and BMI (calculated as weight divided by height squared (kg/m^2^)), BP (including the SBP and DBP), FBG level, and inclusion of triglyceride (TG) data, including esters, total cholesterol (TC), low-density lipoprotein cholesterol (LDL-C), and high-density lipoprotein cholesterol (HDL-C), were collected. The BP, FBG, and blood lipid data of the participants were all automatically measured by special instruments. To ensure the accuracy and stability of the BP data, the participants must keep a calm mind before the BP measurement was performed, and two measurements must be performed. A time interval of 2-3 minutes between the two measurements was required. This study used the second BP measurement as the final measurement. If the difference between the measurement results was too large, the measurement was performed again. Any stroke event that occurred during the 7-year follow-up was marked as an end-point outcome event. All BP records and other variable data were collected and stored in this specialized database system.

### 2.3. Statistical Analysis

Unlike a cross-sectional data analysis, the group-based trajectory model is a more common and effective model for longitudinal data analysis if time-series-like indicator data exist. It is based on the maximum likelihood method to identify clusters of events or outcomes that have a similar progression over time (or age) [31,32]. Changes in the SBP over time were analyzed using a group-based trajectory model that provides three distributions: (1) censored normal (CNORM) for the analysis of censored continuous data, (2) zero-inflated Poisson (ZIP) for the analysis of count data, and (3) binary logistic for the analysis of binary data [33]. Given the continuous measurements of indicator variables in this study, CNORM was used for the analysis to avoid the effects caused by the omission of data. The trajectory analysis was performed using the Proc Traj program in the SAS 9.4 software (SAS Institute, Inc, Cary, NC) program. The number of trajectory subgroups was determined using a combination of four criteria: (a) a comparison of the numerical magnitude of the Bayesian information criterion (BIC) and Akaike information criterion (AIC); (b) a group size such that no less than 5% of the study sample was assigned to one trajectory group; (c) the average posterior probability of group assignment (≥0.7); and (d) the practicality of the analysis, as well as its applicability [23–25]. According to the criteria, three SBP trajectory subgroups were finally identified, as shown in Figure 1. The SBP ranges of the three trajectory subgroups are summarized in Table 2. Next, the participants in the three SBP trajectory groups were characterized at baseline, in which the continuous variables are expressed as mean ± SD and compared using analysis of variance for nonpaired samples of normally distributed parameters, and categorical variables are expressed as the percentage and were compared using the chi-square test, as shown in Table 2. The cumulative risk of stroke among the subgroups of SBP trajectory patterns was analyzed using Kaplan–Meier survival curves, and the survival distributions of the SBP trajectories were compared using the log-rank test, as shown in Figure 2. Finally, the relationship between the SBP trajectory and stroke risk in the three groups was analyzed by a Cox proportional hazards model after adjusting for confounding variables (Table 3). The following is the function of the Cox proportional hazards model.

(1) $$\begin{array}{c} h\left(t|x,z\left(t\right)\right)=h_{0}\left(t\right)\exp\left(\beta z\left(t\right)+\eta^{\prime }x\right)\text{,} \end{array}$$

where *z*(*t*) denotes the time-varying covariate that is invariant for the outcome risk and is represented by the regression coefficient *β*; *x* denotes the time-invariant covariates; *η* is the vector of regression coefficients associated with the vector of fixed covariates *x*; and *h*_0_(*t*) is the baseline hazard function, i.e., the hazard function of the outcome for those participants, with *x* = 0 and *z*(*t*) = 0 [34]. The data analysis was performed using SAS 9.4 software and SPSS 26 software (IBM Corp., Armonk, NY, USA). All statistical tests were considered statistically significant at *P* < 0.05.

## 3. Results

This study utilizes research methodology used by Wang et al., and the description of the methods partly reproduces their wording [29, 30, 32]. In this section, we first grouped the sample based on the SBP using the group-based trajectory model. A second step of survival analysis was performed for each trajectory group using Kaplan–Meier survival curves, and a final step was performed using a Cox proportional hazards model to analyze the association between the SBP trajectory and stroke onset.

### 3.1. Group-Based Trajectory Analysis

Participants with insufficient follow-up and those who dropped out for other reasons were excluded, and 1,451 participants were finally included in the analysis. A total of 159 cases of stroke, according to the definition of stroke indicators, were captured during follow-up. Using the group-based trajectory model, the participants were grouped into three SBP trajectory groups by comparing the BIC and the proportion of the participants within each trajectory group (Figure 1). A total of 33, 105, and 21 participants had a stroke event in the three trajectory groups. Based on the visual description of the SBP trajectory over time, the SBP trajectory groups were named, and they included the following numbers of participants: group 1 was labeled the “low-stable group” (37.6%), group 2 was labeled the “moderate-increasing group” (53.4%), and group 3 was labeled the “high-acutely increasing group” (9%). In addition, the profiles of the SBP for the three trajectory groups are expressed as mean ± SD in Table 2. For the females, 289 participants were assigned to the low-stable group, 516 to the moderate-increasing group, and 70 to the high-acutely increasing group. For the male participants, 231 were assigned to the low-stable group, 302 to the moderate-increasing group, and 43 to the high-acutely increasing group. The baseline characteristics of the participants in each trajectory group are displayed in Table 3. Gender, age, DBP, BMI, and the FBG level were statistically different among the three groups.

### 3.2. Kaplan–Meier Survival Analysis

The Kaplan–Meier curves in Figure 2 demonstrate that a higher SBP was associated with a higher risk of stroke in participants throughout the follow-up time. The results of the log-rank test indicate that the cumulative overall survival was significantly lower in both the moderate-increasing and high-acutely increasing groups than in the low-stable group (*P* < 0.001). Among the three SBP trajectory groups, the high-acutely increasing group exhibited the highest stroke risk of the three groups. The trend in the curves in the first and second groups was essentially the same, but the risk of stroke was higher in the second group than in the first group. That is, the type of SBP trajectory was associated with the risk of stroke over time.

### 3.3. Cox Proportional Hazards Regression Analysis

The association between the SBP trajectory and stroke onset was evaluated based on a Cox proportional hazards model and function analysis. Using the low-stable group as a reference group, model 1 was adjusted for age and sex, and model 2 was adjusted for DBP and BMI on top of model 1. Compared with the low-stable group, the moderate-increasing and high-acutely increasing groups had risk ratios of 1.37 (0.91–2.07) and 1.51 (0.82–2.76) after adjusting the model, and the risk of stroke onset was significantly higher in the high-acutely increasing group than in the other groups (Table 4). The high SBP trajectory was a risk factor for stroke (HR = 3.05, 95% CI: 1.76–5.27, *P* < 0.05), and this relationship persisted even after adjusting for sex, age, DBP, and BMI (HR = 1.51, 95% CI: 0.82–2.76, *P* < 0.05).

## 4. Discussion

Stroke has become the leading cause of death and disability for Chinese citizens, which has created a heavy family and social burden on the country. Stroke has been widely recognized as a preventable and controllable chronic disease, and its risk factors can be controlled to reduce its risk. Among these risk factors, hypertension, as a controllable risk factor, can strengthen the control and monitoring of BP to reduce the occurrence of stroke. SBP can be monitored dynamically to predict the risk of stroke in the population. Suppose there is developmental heterogeneity in the SBP trajectories over time. In this case, it should be theoretically possible to identify people who are at a high risk or clinically significant risk for high BP as early as possible and, beyond that, to distinguish between healthy and unhealthy BP trajectories to investigate risk factors.

One advantage of our study is that it is a large fixed-population longitudinal cohort study with repeated measures of stroke risk factors over a considerable follow-up period. Our study provides a novel description of the longitudinal pattern of hypertension and its association with stroke events among the healthy population in Jiaozuo City using a population-based cohort design. In this study, 1,451 participants who met the criteria underwent four follow-up visits over 7 years and were included in the group-based trajectory model for analysis, yielding subgroups with different trajectories. Three subgroups of participants based on the different trajectories were finally identified: the low-stable group, the moderate-increasing group, and the high-acutely increasing group. Current hypertension guidelines recommend that patients with a SBP/DBP of ≥140/90 mmHg should be routinely defined as being at a high risk for hypertension [35–38]. The SBP of individuals in the low-stable group remains stable and within the normal range; the moderate-increasing group includes individuals whose SBP fluctuates at the border of the normal range with a tendency to increase; and the high-acutely increasing group includes individuals who already have hypertension and also have an SBP that has a tendency to fluctuate and increase. The trends in the moderate-increasing and high-acutely increasing groups suggest that stroke risk factors are changing in an unfavorable direction. As expected, the risk of stroke was significantly higher in the high-acutely increasing group than in the first two groups. In our analysis, clustering groupings indicated that individuals belonging to the high-acutely increasing group had the greatest risk of stroke and that individuals in this group had an urgent need of appropriate antihypertensive treatment. Also, because participants in the moderate-increasing group are on the verge of developing hypertension, they need to pay attention to the BP measurement and control their BP in their daily lives.

SBP trajectories have a stronger ability to detect correlations than individual SBP values at a single point in time [20]. The analysis of systolic trajectories may reflect a population's magnitude of stroke risk. Studies analyzing the association between the SBP trajectory and stroke events have not yet been performed. However, similar results have been obtained in related studies, i.e., those analyzing the relationship between the SBP trajectory and prognostic outcomes of stroke. Lee divided the 1-year SBP into four trajectory groups and demonstrated that patients in the slowly decreasing SBP group and the persistently high SBP trajectory group were prone to poor stroke outcomes [27]. Several studies have investigated the relationship between the SBP trajectory and outcomes in patients with acute cerebral ischemia and acute cerebral hemorrhage. They confirmed that, in the acute phase, a decreasing BP predicted a trend toward good patient outcomes and that longitudinal SBP trajectories exhibited a better risk detection [20, 21, 33]. Consistent with the findings of other studies, the present study confirmed the association of SBP trajectory patterns with stroke risk using a Cox proportional hazards model. Understanding how BP trajectory patterns contribute to the risk of stroke later in life may help to facilitate targeted stroke prevention programs.

It is well known that health indicators for stroke (i.e., age, BP, glucose level, lipid level, and so on) are associated with stroke events. Our study demonstrated that the risk of stroke based on different subgroups was significantly associated with age, sex, BMI, DBP, and the FBG level but was not significantly associated with the TG, TC, LDL-C, and HDL-C levels. The study by Kim et al. concluded that, in addition to high SBP, BMI, and FBG levels, a high TC level is also a risk factor for stroke [39]. Moreover, Ali et al. demonstrated that risk factors, such as gender, low HDL-C level, high LDL-C level, high FBG level, high glycosylated hemoglobin level, and high BP, largely contribute to the development of stroke [40]. In conclusion, the findings of this study in terms of the identification of risk factors were not completely but partially similar to the findings of others. The reason for this may be the geographical differences of the study population.

Hypertension is generally accepted as a modifiable risk factor for stroke. The same was verified in the present study in that the risk of stroke was significantly higher in the high-acutely increasing group than in the other two SBP trajectory groups. The present study bridges the gap and further extends related aspects of research as well as validates the relationship between the SBP trajectory and risk of stroke. A key strength of our study is the systematic analysis of the association between the risk of stroke and SBP trajectories determined by the group-based trajectory model, which has a minimally arbitrary approach to SBP grouping. The study of the SBP trajectory highlights certain advantages and warrants further investigation of its relationship with the risk of stroke in the future. However, the present study has some limitations, as stroke can be divided into ischemic stroke and hemorrhagic stroke. However, this study did not examine the different types of stroke separately, so future studies should refine the study of stroke events to the different types of stroke. There are still some factors that are missing or that were not recorded, such as alcohol consumption and family history, which may also cause some confounding bias, and their effects need to be further investigated. The identification of the type of stroke can be achieved using lightweight deep learning models, which was confirmed by Shelatkar et al. to be an effective diagnostic technique [41]. In addition, various data balancing techniques, such as SMOOTH, can be performed to mitigate the problem of an imbalanced dataset [42].

## 5. Conclusion and Future Work

The Stroke Screening and Intervention Program for People at Risk of Stroke is a project that moves the threshold of prevention forward to the communities and townships through the cooperation between disease control agencies, base hospitals, and primary medical units, and it includes comprehensive stroke risk factor screening for the population. The project can serve as a warning and prevention technique for stroke risk and can continue to be implemented in an in-depth manner.

In conclusion, using the group-based trajectory model may help to elucidate the relationship between the SBP and variation in the SBP and the risk of stroke. The use of this enhanced method may accurately estimate the proportions of the screening population into different SBP trajectories and identify the associated risk factors. This study suggests that there are different SBP trajectories in the health-management population. Each trajectory group has different baseline characteristics and a different level of stroke risk, and a higher SBP trajectory implies that there is a higher stroke risk, suggesting reasonable BP reduction methods and targets for the high SBP trajectory group. In addition, to further improve the accuracy of the analysis, there is a need to refine the types of stroke and to focus on the risk factors for stroke in an integrated manner, which is a plan for our future work.

## Figures and Tables

**Figure 1:** Trajectory groups of SBP (group 1: low-stable group; group 2: moderate-increasing group; group 3: high-acutely increasing group).

**Figure 2:** Risk of stroke in the three SBP trajectory groups (group 1: low-stable group; group 2: moderate-increasing group; group 3: high-acutely increasing group).

**Table 1:** Summary of the advantages and challenges of the SBP trajectories in the literature.

No.	Author	Object	Advantages	Challenges
1	Cederholm et al. [13]	To estimate the risks of fatal/nonfatal coronary heart disease (CHD), stroke, and cardiovascular disease (CVD) according to the SBP in an observational study of patients with type 2 diabetes	The follow-up data captured were based on national registries of morbidity and mortality, which have a high quality and coverage rate	The type and amount of antihypertensive drugs used in the analysis were unclear

2	Portegies et al. [14]	To identify the long-term trajectories of blood pressure in a population-based study and to examine the risk of stroke within those trajectories	(1) The study population was large	(1) The number of stroke subtypes examined was too small
			(2) The data were comprehensive	(2) We did not have information about blood pressure at earlier ages
			(3) The follow-up period was long	

3	Xu et al. [21]	To describe the blood pressure trajectory of patients with ischemic stroke with high blood pressure in the first 7 days of admission and to examine its relationship with clinical outcomes	It highlights the superiority of SBP trajectories over BP levels and single-day variations using a single value	(1) Small sample size
				(2) Changes in blood pressure during the acute phase caused by BP-lowering medications were not considered
				(3) The results may be influenced by selection bias and potential confounding factors
4	Tanaka et al. [27]	The objective of this study was to highlight the heterogeneity of temporal SBP changes in the ATACH-2 trial using GBTM and to analyze the associations with the outcomes of acute intracerebral hemorrhage	The determination of the SBP trajectory grouping was less arbitrary	The results may not be totally applicable to lobar ICH patients because of the low proportion of lobar ICH in ATACH-2
5	Lee et al. [28]	To describe the patterns of BP changes up to 1 year after ischemic stroke using group-based trajectory models and to explore the associations between the BP trajectory group and poststroke cardiovascular outcomes	The results of the study are robust	(1) The sample selection is biased
				(2) The generalizability of the results of the study to the entire population of patients with stroke may be limited
6	Wang et al. [29]	To investigate whether the long-term trajectories of a high SBP can further predict the risk of all-cause death in Chinese adults	Large sample size	(1) A specific classification of the causes of death is not given
				(2) The follow-up period was relatively short for SBP trajectory patterns
7	Kim et al. [30]	To explore the relationship between different trajectory groups and stroke characteristics and the risk of subsequent recurrent vascular events	(1) This is the first study to apply group-based trajectory models to investigate the heterogeneity in SBP trajectories during the acute stroke period	(1) An analysis of increasing antihypertensive drugs, as well as other influencing factors, was not performed
			(2) The findings may be generalizable to patients with acute stroke in Korea	(2) Studies may have limited generalizability

**Table 2:** Follow-up circumstances of the SBP trajectory groups.

Groups	1	2	3	4
Low-stable group	123.78 ± 10.60	122.75 ± 12.49	123.28 ± 9.75	124.50 ± 11.72
Moderate-increasing group	134.84 ± 13.45	145.07 ± 15.62	138.15 ± 10.87	145.54 ± 15.65
High-acutely increasing group	144.53 ± 19.78	176.23 ± 19.79	160.49 ± 20.89	170.26 ± 20.86

**Table 3:** Baseline characteristics of the SBP trajectory groups.

Variable	Low-stable group	Moderate-increasing group	High-acutely increasing group	*P* value
*N*	520 (35.84%)	818 (56.37%)	113 (7.79%)	
Sex (male)	231 (44.42)	302 (36.92)	43 (38.05)	0.0119
Age	55.98 ± 9.49	61.13 ± 9.51	66.8 ± 9.23	<0.0001
BMI	24.54 ± 3.19	5.45 ± 3.42	25.88 ± 3.84	<0.0001
SBP	123.78 ± 10.6	134.84 ± 13.45	144.53 ± 19.78	<0.0001
DBP	79.19 ± 7.75	83.64 ± 10.33	87.28 ± 12.35	<0.0001
FBG	5.35 ± 1.39	5.62 ± 1.54	5.44 ± 1.34	0.0057
TG	1.60 ± 1.01	1.73 ± 0.97	1.69 ± 0.79	0.0922
TC	4.66 ± 1.16	4.77 ± 1.24	4.95 ± 1.08	0.0541
LDL-C	2.65 ± 0.87	2.62 ± 0.84	2.67 ± 0.89	0.8401
HDL-C	1.50 ± 0.69	1.51 ± 0.64	1.48 ± 0.64	0.8884

BMI: body mass index; SBP: systolic blood pressure; DBP: diastolic blood pressure; FBG: fasting blood glucose; TG: triglycerides; TC: total cholesterol; LDL-C: low-density lipoprotein cholesterol; HDL-C: high-density lipoprotein cholesterol.

**Table 4:** Hazard ratios and 95% confidence intervals for stroke for the three SBP trajectories.

	Hazard ratio (95% CI)			*P*
	Model 1	Model 2	Model 3	
Group 1	1	1	1	<0.05
Low-stable group				
Group 2	2.06 (1.39–3.04)	1.60 (1.07–2.38)	1.38 (0.91–2.07)	<0.05
Moderate-increasing group				
Group 3	3.05 (1.76–5.27)	2.05 (1.16–3.64)	1.51 (0.82–2.76)	<0.05
High-acutely increasing group				

## Data Availability

The data used to support the findings of this study are available from the corresponding author upon request.
